# A Method for Evaluating the Quality of Mathematics Education Based on Artificial Neural Network

**DOI:** 10.1155/2022/6976654

**Published:** 2022-08-12

**Authors:** Fuli Bao, Chong Wang

**Affiliations:** ^1^Department of Ideology and Politics, Inner Mongolia Vocational and Technical College of Communications, Chifeng 024005, China; ^2^School of Mathematical Sciences, Daqing Normal University, Daqing 163712, China

## Abstract

Teaching quality evaluation (TQE) is an important link in the process of school teaching management. Evaluation indicators and teaching quality have a complicated and nonlinear connection that is influenced by several variables. Some of these drawbacks include too much subjectivity and unpredictability, difficulty in defining index weights, sluggish convergence, and weak computer capacity. The current assessment techniques and models have these issues as well. This research uses an ANN model to assess the quality of mathematics instruction at colleges and universities (CAU) in order to address the challenging nonlinear issue of TQE and completes the following tasks. (1) The background and significance of TQE research are analyzed, and the domestic and foreign research status of TQE and neural network is systematically expounded. (2) The technical principle of DNN is introduced and the DDAE-SVR DNN model is constructed, and then, the evaluation index system of mathematics teaching quality is constructed. (3) The DDAE-SVR DNN model is put out as a potential alternative. The Adam method is used in the unsupervised training process to dynamically modify the learning step size for each training parameter. The spatial properties of the original data may be modified several times such that the reconstruction can be completed after many hidden layers have been applied. Data essentials such as precision, accuracy, and consistency are prioritized above all other considerations when generating the final product. Unsupervised prediction uses SVR and maps the complicated nonlinear connection into high-dimensional space in order to attain linearity in low-dimensional space, which is the goal of the supervised prediction process. The usefulness and benefits of the model provided in this research in the mathematics TQE may be verified by tests including the use of the TQE dataset and comparisons with other shallow models.

## 1. Introduction

Since our country's reform and opening up, we have seen remarkable growth in every sector. Every day, the need for skills grows, and the quality of a country's talent pool is linked to its overall competitiveness in the global marketplace [1]. The popularization of higher education is also related to the cultivation and reserve of talents. In order to narrow the gap between the educational level of our country and foreign countries and improve the quality of the people in an all-round way, our country has expanded the scale of college enrollment since 1999. Since the first full implementation of online enrollment in 2002, as of 2003, the number of undergraduate and junior college students in general CAU nationwide has exceeded 10 million [2]. Quality teaching is a critical component of a school's overall administration, and it serves as a crucial indication for determining whether or not a school is succeeding. Teachers' TQE enables school leaders and managers comprehend the extent to which teaching goals have been met, as well as thoroughly and properly grasp the school's teaching work and enhance the quality of teaching [3]. TQE related to teaching quality will also become a very important task. TQE constitutes the basis of teaching activities in CAU and is the basic link to ensure the quality of personnel training in CAU. There are a number of ways in which the TQE may be used to improve teaching quality and promote change, and it has a significant impact on overall educational quality. However, because teaching is a kind of mental labor, there is no fixed process, and the TQE system often contains nonquantitative factors, which constitutes the complexity and difficulty of TQE. The teaching process includes teaching and learning. A teacher's TQE is much more complicated than the quality evaluation of a product [4]. There are numerous aspects that go into the teaching process, which is a two-way street between the instructor and learner. There is a wide range of topics to consider when assessing a teacher's ability to instruct effectively. How to establish a scientific and reasonable TQE system so that it can evaluate the teaching quality objectively and fairly is a very meaningful subject. According to reference [5], the integration of information technology into higher education, the modernisation of educational material, and the general development of the quality of higher education should be a primary goal of this research. It is imperative that we tackle the challenge of evaluating the teaching quality at CAU in a fair and accurate manner in order to further the higher education reform and enhance CAU's teaching goals and quality. That is why studying ways to improve teaching quality at CAU has emerged as an essential research issue in the effort to make education and training more scientific and standardized. An ANN is a nonlinear system made up of a large number of computational neurons arranged in layers that may be altered in many ways. Large-scale parallel processing, self-organizing white learning, and nonlinear capabilities make it an attractive alternative to traditional computing methods in many situations. There are many applications where ANN may be used that standard techniques and models cannot, and the results are excellent. ANN is a mathematical model for processing computation. Gradient-descent correction is used in BPNN to rectify the error signal produced during forward propagation until the accuracy objective or the number of iterations is satisfied [6]. As time went on, researchers discovered that every closed interval continuous function could be approximated by a BPNN hidden layer, meaning that any three-layer BPNN could complete any *n*-to-*m*-dimensional mapping [7]. A deep learning structure called a multilayer perceptron, which has numerous hidden layers, may be utilized to handle increasingly difficult nonlinear problems [8]. Layer-by-layer unsupervised greedy training using DBN is being proposed by researchers. Multiple restricted Boltzmann machines (RBM) in sequence stack a DBN into a deep structure in the method, which offers promise for tackling optimization difficulties connected to deep structures. A deep structural model based on a multilayer autoencoder is presented [9, 10]. There was a spike in DNN research when the findings were released, and neural network models' number of layers and size have both increased dramatically since then. A complete assessment of instructional activities is thus necessary, and this study suggests the DDAE-SVR DNN model as a solution for the limitations of the current methodologies and models. In order to improve the teaching quality to promote the reform and development of CAU, establish a scientific TQE system in CAU to strengthen the teaching management of CAU.

## 2. Related Work

For a long time, many educators in our country have been constantly studying how to construct an objective and scientific TQE system and improve it. However, Western nations began sooner than my country and experienced some successes, which led to the development of more effective approaches such as multiple intelligences' theory and constructivism. Taylor assessment model was also developed [11]. Since the concept of TQE was formed in the second half of the 19th century, it can be divided into five stages: examination, test, description, reflection, and construction according to the characteristics of each period [12]. The initial TQE exists in the form of examinations, and the results are largely influenced by teachers' subjective judgments. In the 1930s, in order to strengthen the objectivity and rationality of evaluation, educators put forward the term test and formed the concept of educational evaluation. At this time, the achievement of educational goals is evaluated through the description of students' learning behavior. It can be said that this is a breakthrough development of pedagogical evaluation methods. Since the rapid economic growth of China has supplied the necessary conditions and materials for the development of Chinese education, a wide range of theoretical studies into TQE has been conducted. There have been several teaching assessment methods presented by educators throughout the years. Reference [13] established a TQE system using fuzzy algorithms to improve the quality evaluation of schools. It can also conduct self-evaluation in stages according to the actual situation of students. Reference [14] used the analytic hierarchy process (AHP) to quantitatively evaluate the teaching quality of CAU and formed a corresponding evaluation system. Reference [15] constructed a set of teaching quality monitoring system based on the concept of “people-oriented, three-dimensional integration.” The “people-oriented” in the system mainly refers to teachers and students-oriented, while “three-dimensional” refers to the top-level dimension (school), the middle dimension (second-level college), and the basic dimension (teacher). Reference [16], under the guidance of the national dual innovation and development strategy, adopts the mathematical fuzzy AHP and introduces diversified evaluation methods to change the supervision function and solve the problems existing in the TQE. Reference [17] designs the implementation process of the blended teaching model and builds a blended TQE model according to the teaching results, which has achieved good results in practical applications. To guarantee that the quality of teaching is maintained, a variety of types of higher teaching assessment have been established across the globe and play a more active part in the teaching process. Because it is a nonlinear classification issue, assessing the quality of higher education instruction is complex. So while developing a TQE system, it is important to identify the most fundamental elements that may immediately represent the quality of teaching. With the development of computer technology and information technology, many scholars have adopted a mathematical model to directly establish a TQE system. The content and methods of assessment are also diverse among CAUs because of their differing views on teaching excellence [18]. Reference [19] applied a multilevel evaluation model of type II fuzzy sets to the performance TQE. Reference [20] applied AHP and neural network in the TQE model. Reference [21] developed a TQE model by combining the fuzzy AHP with the fuzzy comprehensive assessment approach, giving higher education administrators another instrument for raising the level of teaching quality. Reference [22] applied the TOPSIS method of multiattribute decision-making in TQE for research. Reference [23] uses BPNN and related theories to formulate the evaluation index system, constructs an effective computer graphics TQE model, and uses this model to evaluate the actual teaching situation of related courses. Reference [24] proposed an optimized BP algorithm, and the results after applying it to actual training show that the evaluation model established by this algorithm has fast convergence speed and high accuracy and has broad application prospects in teaching evaluation problems in higher education. Reference [25] combined AHP and neural network, combined the advantages of the two, added a screening process in the evaluation, and finally got the AHP-BPNN evaluation model. Using the PSO method, Reference [26] establishes a complete model for evaluating college professors' teaching quality by optimizing a neural network and finding the global optimum network parameters. By using ANN theory in TQE, not only are the difficulties of qualitative and quantitative indicators in a complete evaluation index system solved but also are the challenges of establishing complicated mathematical models and analytical expressions inside a conventional evaluation process resolved. It also reduces the impact of human error on the assessment process, resulting in more precise and effective findings. The TQE model developed by neural network theory is a useful tool for TQE.

## 3. Method

### 3.1. Deep Neural Network Theory

#### 3.1.1. Deep Neural Networks

DNN is a deepening structure of ANN, and its network structure contains multiple hidden layers, which can better obtain learning features from input sample data. Since the 1940s, a large number of scholars and research institutions have devoted themselves to the research of ANN models, but most of the models are shallow models containing only one hidden layer, for example, three-layer BPNN model, maximum entropy model, traditional Markov model, and conditional random field. The hidden layer of the model converts the original data information input into the network through the input layer into the feature space required by a specific problem or target, which is the key to information processing. It is mainly used in classification, regression, pattern recognition, and other problems. However, since the shallow neural network model has only one hidden layer, its computing power, efficiency, and modeling ability will be limited in the face of high-order complex nonlinear functions. Therefore, the DNN that contains multiple hidden layer neural networks to better obtain the feature vectors of the sample data has become the focus of researchers. The training of neural network models with deep structures is not easy, and the mappings produced by deep models are nonconvex functions, which are extremely difficult to study theoretically. The proposal of DBN and unsupervised greedy layer-by-layer training algorithm has opened up the research wave of DNN model. The multiple hidden layers of the DNN model have good feature learning ability, and the acquired data features can well represent the nature of the data. In the training process of the DNN model, the unsupervised greedy layer-by-layer learning algorithm initializes the deep structure layer by layer and then uses the supervised algorithm to fine-tune the model parameters. This method overcomes the problems encountered in the training process of traditional models and improves the efficiency of DNN models. By designing multiple hidden layers, the DNN performs multiple feature space transformations on the sample data, obtains good data feature vectors, and realizes the fitting of complex nonlinear mapping relationships. The arrival of the era of big data has provided many datasets for the training of DNN models, such as ImageNet image recognition dataset and Project Gutenberg language model dataset.

#### 3.1.2. Basic Model of Deep Neural Network

DNN may be implemented in a variety of ways. There are two primary models discussed here: the RBM model and the autoencoder model.

1. Autoencoder model: in 1986, the idea of an autoencoder was initially put out. It is an algorithm that is used mostly for data reduction and feature extraction. There are two networks that make up the autoencoder: one to encode and one to decode. There are three layers to this model. Error propagation utilizing the BP technique is the underlying premise, and network weights and thresholds are constantly updated to recreate the original data. In order to generate a copy of the original data, the final output data are trimmed. First, the encoder network transforms the input data, such as reducing the number of dimensions in the input data. By first synthesizing the original input data using a decoding network and then using an error function to assess how much of the original input data is being incorrectly reproduced, this may be done. In order to provide an output that is as close to the input as feasible, an autoencoder must find an approximation identity function. For example, if the input data feature vector is *h* in the hidden layer and the output feature vector is *y*, the decoder from the middle hidden layer to the output layer and the autoencoder from the input data feature vector to the middle hidden layer are used, respectively, to decode *x* and encode *h*, mapped using the following mathematical expression:

(1) $$\begin{array}{c} h=f\left(x_{i}\right)=A_{f}\left(W_{f}x_{i}+p_{i}\right),\\ y=g\left(h_{i}\right)=A_{g}\left(W_{g}x_{i}+p_{j}\right), \end{array}$$

where *f* and *g* are the encoding function and decoding function, respectively; *A*_*f*_ and *A*_*g*_ are the activation functions of encoding and decoding, respectively, which are generally nonlinear functions; *W*_*f*_ and *W*_*g*_ and *p*_*i*_ and *p*_*j*_ are the weight matrix and threshold value matrix of the network, respectively.

It is common for autoencoders to use the gradient descent approach in order to fine-tune layer weights and thresholds in order to reduce the amount of error in reassembling the original input data. MSE or cross-entropy loss (CEL) functions are often used as the cost function, and the expression is as follows:

(2) $$\begin{array}{c} L\left(x,y\right)=\frac{1}{n}\overset{n}{\underset{i=1}{\sum }}{\left(y_{i}-x_{i}\right)}^{2},\\ L\left(x,y\right)=\frac{1}{n}\overset{n}{\underset{i=1}{\sum }}x_{i}\log\left(y_{i}\right)+\left(1-x_{i}\right)\log\left(1-y_{i}\right). \end{array}$$

(2) RBM model: the RBM model is an improvement of the BM. An undirected two-layer graph model is used. Nodes between the visible and hidden layers are connected by the RBM model, while all other nodes are left unconnected. Boltzmann machine units are connected only between neighboring layers, and the cross-layer unit is not connected to the same layer unit. RBM's bipartite graph model assumes that the units in its visible and hidden layers may be distributed arbitrarily exponentially, *v*_*i*_ ∈ {0, 1}, *h*_*j*_ ∈ {0, 1}, where (*i* = 1, 2, 3, ⋯, *n*; *j* = 1, 2, 3, ⋯, *m*). To determine the RBM model, we only need to get *θ* = {*w*_*ij*_, *a*_*i*_, *b*_*j*_}, where *w*_*ij*_ is the connection weight between the visible layer and the hidden layer unit and *a*_*i*_ and *b*_*j*_ represent the visible layer and the hidden layer, respectively, offset of the unit. For a given set of states (*v*, *h*), the energy formulation of the RBM is as follows:

(3) $$\begin{array}{c} E\left(\left.v,h\right|\theta \right)=-\overset{n}{\underset{i=1}{\sum }}a_{i}v_{i}-\overset{m}{\underset{j=1}{\sum }}b_{j}h_{j}-\overset{n}{\underset{i=1}{\sum }}\overset{m}{\underset{j=1}{\sum }}v_{i}w_{ij}h_{j}. \end{array}$$

The joint probability distribution (*v*, *h*) of the visible layer unit and the hidden layer unit in a specific state may be determined by exponentiating and regularizing the energy function.

(4) $$\begin{array}{c} P\left(\left.v,h\right|\theta \right)=\frac{e^{-E\left(\left.v,h\right|\theta \right)}}{Z\left(\theta \right)},\\ Z\left(\theta \right)=\underset{v,h}{\sum }e^{-E\left(\left.v,h\right|\theta \right)}. \end{array}$$

This yields the marginal distribution of visible and buried layer unit sizes, with *Z*(*θ*) serving as a normalization factor. By using a greedy learning technique to train several RBMs, the DBN model may be thought of as a Bayesian probabilistic generative model.

### 3.2. DDAE-SVR Deep Neural Network Model

#### 3.2.1. Deep Denoising Autoencoder

DDAE is a typical neural network architecture consisting of many DAE layered; therefore, it includes several hidden layers. In order to avoid overfitting during the training process, after unsupervised training, a model with strong robustness and generalization emerges from the DAE's addition of noise to the original input dataset. Dataset denoising is the first step in training a deep noise reduction autoencoder. Input nodes are often set to 0 with a specified frequency as a generic processing strategy. Once the dataset has been denoised, it is sent into the first DAE to perform the data feature modification. The output of the first DAE's hidden layer is utilized as the input feature vector for the second autoencoder's second autoencoding layer. Until all DAEs have been trained, the output of the preceding DAE's hidden layer is utilized as the input feature vector for the succeeding DAE. To put it another way, when the original data has been denoised, the data feature conversion is completed by training each hidden layer one by one, unsupervised. An error function may be used to calculate the difference between a reconstructed dataset and the original dataset. In order to complete the reconstruction of the original input dataset, error propagation and option weight and threshold adjustments are made using BP in order to lower the overall error. As an unsupervised training approach, this portion of the DDAE introduces the Adam method. A classification or regression prediction may be improved by changing the parameters of a classifier or predictor in the DDAE's actual output layer, which is a virtual representation of the DDAE's virtual output layer neurons.

#### 3.2.2. Support Vector Regression

SVM is a machine learning technique based on statistical theory. As a decision surface, a categorization hyperplane is needed to separate positive and negative occurrences of the same notion more effectively. Classification, pattern recognition, and return are some of the most common uses for it. Some of the advantages of SVMs in dealing with complex nonlinear issues and high-dimensional pattern recognition may be attributed to the use of a limited number of learned patterns. It is difficult to represent in mathematical analysis the complicated nonlinear connection between the evaluation indicators and the TQE findings at CAU since there are numerous indications of teaching quality assessment. Although SVR has an excellent nonlinear function fitting ability, this issue may be solved by using it. As a result, in order to assess and forecast teaching quality, the output layer of the DNN model is predicted using SVR in this chapter. In multidimensional space, the SVR is divided into linear regression and nonlinear regression, which are then combined. SVR's nonlinear regression is the emphasis of this part, since the quality of CAU's instruction is a complex nonlinear problem to solve. To achieve a linearization connection comparable to the low-dimensional space, SVR uses nonlinear regression to transfer a complicated nonlinear relationship onto a high-dimensional space. A nonlinear mapping function should be used to map the dataset *S* to a high-dimensional space, and the linear regression characteristics of the feature space *H* should be taken into consideration when setting up the mapping function for the dataset *S* that cannot be linearly separated in the original space *R*^*n*^. As a result, to describe nonlinear issues linearly, do linear regression in *H* first in the feature space before returning to *R*^*n*^, the original space. Given a kernel function *K*(*x*_*i*_, *x*) = (Ø(*x*_*i*_), Ø(*x*)), the representation of the built nonlinear function is as follows:

(5) $$\begin{array}{c} f\left(x\right)=\overset{S}{\underset{i=1}{\sum }}\left(\alpha_{i}-\alpha_{i}^{*}\right)K\left(x_{i},x\right)+b. \end{array}$$

#### 3.2.3. DDAE-SVR Deep Neural Network Model

Low-level noise reduction due to the restricted computational and modeling capability of the shallow neural network model, the DDAE-SVR DNN model uses an unsupervised training layer and SVR as a prediction output layer to solve complicated nonlinear issues or analyze large-scale datasets. Instead of relying on techniques like first- and second-order moment estimation and second-order moment estimation, unsupervised training utilizes the Adam optimization methodology to boost convergence and processing power. After the input dataset has been denoised using a DDAE, the model is trained using unsupervised layer-by-layer learning. Make sure the unsupervised training data is as close to the original dataset as possible when generating feature vectors for the original input. An input feature vector created from the model's final output layer is fed into SVR as a predictor, and SVR is used as a predictor for the final output layer. The DDAE-SVR DNN model's two most important features are as follows.

1. For the DDAE-SVR DNN model, the original input data will be weighted according to a set percentage before being fed into the unsupervised layer-by-layer training technique to prevent overfitting. The characteristics have been set to 0 in order to improve the model's robustness and generalizability. Deep noise reduction autoencoders are mostly used during the unsupervised training phase of the learning process. Using the result of the first DAE as an input feature vector, the data from the input layer is sent into the second DAE for training, and so on. Each DAE becomes a hidden layer of DDAE once it has been trained. Iterate the Adam algorithm until a specified accuracy or number of iterations is attained, or until a specific number of iterations has been completed
2. The final output layer of the DDAE-SVR DNN model uses the feature vector from the DDAE's final hidden layer as an input feature vector for the supervised fine-tuning procedure. SVR, a supervised algorithm, serves as the predictor in the final output layer. Predictive accuracy and efficiency are improved in this supervised prediction process by tuning parameters relevant to SVR

### 3.3. DDAE-SVR DNN Mathematics Education Quality Evaluation Model

It is possible to extract characteristics from the original sample data using the deep-structured neural network model's many hidden layers. To solve complex nonlinear issues or deal with the in-depth structure of large datasets, the neural network model introduced in this chapter is used by CAU. This is a normalized evaluation index sample data collection, and we have *n* samples in it. Assuming *W* is the weight matrices of the DDAE model's various layers, *p* is the threshold matrices, and *Ø* is the DDAE model itself. As a result, once *Ø* processes the incoming dataset, its expression is as follows.

(6) $$\begin{array}{c} \theta =\phi \left(WX+p\right), \end{array}$$

where *θ* represents the output feature vector of the deep noise reduction autoencoder model, *θ* is input into the SVR model for evaluation and prediction, and *f* is used as a function of the SVR model; the expression is as follows.

(7) $$\begin{array}{c} y_{d}=f\left(\theta \right). \end{array}$$

This chapter recommends that the evaluation sample data be divided into two sets: one for training and one for testing. The model is then trained using the training dataset. The test dataset is used to verify the model's performance in the TQE issue after developing a stable and optimal model.  Figure 1 depicts the DDAE-SVR DNN model's flowchart for assessing the validity of the mathematical reasoning.

### 3.4. Mathematical TQE Index System

Multilevel and multiobjective optimization is the name of the game when it comes to the CAU TQE. As a result, the assessment indicators should not only represent the teaching process in its whole and objectively but also limit the number of evaluation indicators as much as feasible. Both “teaching” and “learning” are important concepts in classroom discussions. Both the students' and the teachers' evaluation indicators are based on input from those who are most acquainted with the teaching process and its distinctive features, namely, the students' and the teachers' evaluation indicators from the teaching supervision group. Students' evaluations of instructors might best represent the issues with educational activities since they serve as the major body of learning. The evaluation indicators are shown in Table 1.

Since the input data of the network has different dimensions and physical meanings, the input features have different numerical ranges and the numerical ranges between different features vary greatly, so the sample data is normalized and preprocessed. After normalization, the data is converted into [0, 1] to reduce the difficulty of weight correction due to the large variation of the input value. On the other hand, the excitation function of the BPNN is a sigmoid function, and the derivative of the function changes in [0, 1] in a large definition domain. The normalization of the sample data helps the network to converge as soon as possible, thereby improving the computational efficiency of BPNN. The method used in this article is as follows:

(8) $$\begin{array}{c} x_{i}=\frac{x-x_{\min}}{x_{\max}-x_{\min}}, \end{array}$$

where *x*_max_ represents the maximum value in the data, *x*_min_ represents the minimum value in the data, and *x* and *x*_*i*_ represent the data before processing and the output data after processing.

## 4. Experiment and Analysis

### 4.1. Dataset Sources and Evaluation Indicators

This research uses data from a university's educational administration system to compile an assessment dataset for math courses taught between 2012 and 2018, totaling 1685 samples. Data gathered from students' evaluations of a teacher's teaching process is utilized as an input value in the assessment model. In order to ensure model verification, the comprehensive score is employed as the model's goal predicted output value based on the numerous lecture recordings of teaching supervision group instructors. A total of 1520 sample data were collected after analyzing the dataset and removing the data with high, low, and inconsistent evaluations. The resultant data samples are then subjected to normalization preprocessing.

As part of the DDAE, a new method known as the Adam algorithm is implemented, which minimizes output data error while preserving as many of the original data's key properties as possible. In order to increase the model's accuracy in making predictions, the key SVR parameters are tweaked in the supervised output layer. Performance comparison measurements are used to compare this model to other shallow models. Model assessment and prediction accuracy are evaluated using MAPE, MSE, SMAPE, and RMSE in this chapter's DDAE-SVR DNN model, which gives more advantages than other models in terms of mathematical quality evaluation. These are the formulas they use. This includes test data's sample size (*n*), actual value of the data (*p*_*i*_), and its model's anticipated value (*r*_*i*_).

(9) $$\begin{array}{c} \text{MAPE}=\frac{1}{n}\overset{n}{\underset{i=1}{\sum }}\left|\frac{r_{i}-p_{i}}{r_{i}}\right|,\\ \text{MSE}=\frac{1}{n}\overset{n}{\underset{i=1}{\sum }}{\left(p_{i}-r_{i}\right)}^{2},\\ \text{SMAPE}=\frac{1}{n}\overset{n}{\underset{i=1}{\sum }}\frac{\left|r_{i}-p_{i}\right|}{\left(\left|r_{i}\right|+\left|p_{i}\right|\right)/2},\\ \text{RMSE}=\sqrt{\frac{1}{n}\overset{n}{\underset{i=1}{\sum }}{\left(p_{i}-r_{i}\right)}^{2}}. \end{array}$$

### 4.2. Model Parameter Analysis

To get the most out of a TQE model, it is necessary to identify the model's important parameters. For the time being, much of it takes the shape of experiments. Throughout the experiment, model parameters are regularly changed to improve computing capacity and forecast accuracy and to discover the greatest possible combination of model parameters. In order to improve the model's accuracy in making predictions about the quality of the teaching process, this section employs both unsupervised learning training and supervised prediction output.

1. There are a variety of methods utilized in the neural network model's training phase, including the gradient descent and RMSProp techniques. Gradient descent has become a common optimization technique for neural network models with several hidden layers because of its slow convergence as it approaches the lowest value and its ease of slipping into the local minimum value. As a result, the Adam method is introduced in this part as an optimization strategy for the DDAE-SVR DNN model's unsupervised learning training. The Adam method dynamically adjusts the learning step size of each parameter using first- and second-order moment estimations of the gradient. Because of this, the settings are more or less constant between iterations. It is the MSE function and gradient descent that is used to figure out the error between unsupervised training output and input data in the DDAE-SVR DNN model, assuming there are three hidden layers and 20 neurons in each hidden layer. There are four optimization methods used to train and compute the error: the RMSProp algorithm, momentum algorithm, and Adam algorithm. Their error change curves are given in Figure 2. According to Figure 2, the GD and momentum algorithms have been decreasing in efficiency, although at a slow pace and with an increasing number of rounds. Figure 2 illustrates a slow convergence rate. In the first 500 iterations, error in feature vectors generated by RMSProp and Adam algorithms may be quickly decreased utilizing these techniques. Regardless how many iterations are performed, the convergence of error tends to stay flat. The Adam algorithm is used as the optimal approach for unsupervised learning training because it is the most successful at recreating the original input data

Determine how many hidden layers a DNN model needs, and take into account the size of its evaluation dataset. The hidden layer has a total of 20 neurons and may have anywhere from 2 to 5 hidden layers. Unsupervised learning training uses the Adam algorithm as an optimization tool. The evaluation sample dataset is used to train the DDAE-SVR DNN model. We trained an unsupervised DDAE, and the resulting reconstructed feature vector differed significantly from the original input dataset, as seen in Figure 3. With more repetitions of training, it can be seen that there is a decrease in the error between output data and original input data. With a constant number of repetitive training, the error rises with each additional hidden layer. So, after unsupervised training, the DDAE-SVR DNN model with two hidden layers minimizes error between the reconstructed output data and the original input data.

The DDAE-SVR DNN model uses a range of 21 to 25 neurons in each hidden layer to arrive at the final number. Unsupervised learning is used in conjunction with two hidden layers and an optimization strategy in the Adam approach to build the model. Each time an evaluation sample dataset is introduced into the model during training, the hidden layer's number of neurons is modified to account for the changes. By training the DDAE unsupervised, the DDAE is able to rebuild the error curve between output data and the original input data, as illustrated in Figure 4. The error between the reconstructed output data and the original input data decreases while the number of neurons in the hidden layer stays constant. The more neurons in the hidden layer there are, the more effective iterative training is at correcting this error. DDAE-SVR DNN uses 25 hidden layers to provide output data with the lowest feasible error margin when compared to original input data.

(2) Final hidden layer neurons may be acquired using DDAE-SVR DNN model's unsupervised learning and training approach, which reduces the error between the output data reconstructed from final hidden layer and original input data. For the model prediction output layer, a feature vector is utilized as an input. The model's final output prediction layer evaluates and predicts the TQE using the SVR prediction period. In terms of SVR performance, error penalty coefficient *v* and kernel function type are two of the most important considerations to make. This model's complexity and risk may be changed by adjusting its mistake penalty coefficient. In the model, the number of support vectors and training errors is determined by the variable *V*, which has a range of (0, 1). The distribution of sample data in high-dimensional space is controlled by the kernel function type. As a result, improving SVR's prediction efficiency and accuracy requires tweaking these three key parameters. Kernel function types include linear, polynomial, sigmoid, and radial basis functions; the error penalty coefficient range is set at [1, 10], *v* = 0, in light of the sample dataset's size. Unsupervised training is the only way to uncover the last layer of information. As part of the DDAE-SVR DNN model's prediction assessment, the output feature vector is utilized as an input feature vector for DDAE-SVR DNN model's output feature layer. The SVR is then used to evaluate prediction accuracy.  Figure 5 illustrates this. The MAPE error of the evaluation prediction increases as the error penalty coefficient increases, as can be shown in the figure. This is true regardless of the SVR kernel function employed as the error penalty coefficient. Due to the short sample size of the assessment dataset, an increase in the penalty coefficient will result in an excessive penalty, which in turn will raise the MAPE. Using a polynomial function as a kernel function rather than the other three functions improves the SVR model's prediction accuracy; hence, the error penalty coefficient for the SVR model has been set to 1

*v*, the training error parameter, is controlled by a polynomial kernel function, and an error penalty coefficient of 1 is used in this DNN model. The optimal value for [0.1, 1] may be used to regulate the number of support vectors and training error. We use a feature vector from the model's final hidden layer neuron that was trained without supervision to acquire the input feature vector for SVR. MAPE and MSE values both exhibit a decreasing and subsequently increasing pattern with respect to time as seen in Figure 6. If *v* is 0.3, this chapter's model has the least prediction error and the highest accuracy.

### 4.3. Comparison with Other Models

According to this chapter's hypothesis, the DDAE-SVR DNN model provided in this chapter has a better TQE than other models; hence, this chapter optimizes the model's parameters. For comparison, three models of the conventional BPNN, SVM, and adaptive BPNN were built. To train and evaluate the model, input the evaluation sample dataset and denormalize the prediction and evaluation outcomes. Comparisons are made using performance measures like MAPE and MSE.  Table 2 shows the comparing findings. There are several advantages to this neural network model; however, it takes longer to train than other neural network models, as seen in this table. Thus, this paper's model has been shown to be successful.

## 5. Conclusion

High-quality talent is the primary aim of higher education, and teaching quality is an essential way of achieving this goal. The TQE at CAU is a crucial strand in the web of educational administration. Every day, college professors are evaluated on their ability to teach in an objective and fair manner using objective, scientific methods. It is a useful tool for assessing how well the school's teachers are doing their jobs. In order to increase the quality of instruction, managers may learn from teachers' classroom activities how well their teaching strategies are working in practice. However, TQE is mostly a nonlinear classification problem. It is a multifactor complex system with qualitative and quantitative indicators. Because the indicators are multilevel and complex, it is hard to put a finger on it using a predetermined mathematical model. TQE makes use of a number of well-established assessment techniques, including the weighted mean method, AHP, and the fuzzy comprehensive judgment approach, among others. Although some achievements have been achieved, there are still many defects, such as lack of self-learning ability, and it is difficult to make accurate evaluations. When determining the weight of each evaluation index, it is often estimated by experience, which leads to the subjective evaluation and cannot solve the problem well. Therefore, this paper builds a DDAE-SVR DNN model to evaluate the quality of mathematics teaching and completes the following tasks. (1) The background and significance of TQE research are analyzed, and the domestic and foreign research status of TQE and neural network is systematically expounded. (2) The technical principle of DNN is introduced and the DDAE-SVR DNN model is constructed, and then, the evaluation index system of mathematics teaching quality is constructed. (3) The DDAE-SVR DNN model is put out as a potential alternative. The Adam method is used in the unsupervised training process to dynamically modify the learning step size for each training parameter. The spatial properties of the original data may be modified several times such that the reconstruction can be completed after many hidden layers have been applied. Data essentials such as precision, accuracy, and consistency are prioritized above all other considerations when generating the final product. Unsupervised prediction uses SVR and maps the complicated nonlinear connection into high-dimensional space in order to attain linearity in low-dimensional space, which is the goal of the supervised prediction process. The usefulness and benefits of the model provided in this research in the mathematics TQE may be verified by tests including the use of the TQE dataset and comparisons with other shallow models.Лысенко

## Figures and Tables

**Figure 1:** Flowchart of DDAE-SVR DNN model for evaluating mathematical quality.

**Figure 2:** Comparison of training errors of different optimization algorithms.

**Figure 3:** Comparison of layer errors of different hidden layers.

**Figure 4:** Selection of different numbers of neurons in the hidden layer.

**Figure 5:** Selection of kernel function and penalty coefficient.

**Figure 6:** MAPE and MSE variation for different parameters *v*.

**Table 1:** Mathematical TQE index system.

Index	Label
Lectures on time, dedicated to work	B1
Full of energy, serious, and contagious in class	B2
Openly listen to opinions and improve teaching methods and content	B3
Treat students equally	B4
Emphasis on basic theoretical knowledge and teaching of methods	B5
Difficulties are highlighted, and the details are appropriate	B6
Combining theory with practice	B7
Expand the frontiers of disciplinary knowledge	B8
Teaching students according to their aptitude and stimulating interest	B9
Explain clearly and logically	B10
Effective use of multimedia aids in teaching	B11
Satisfied with the teacher's attitude and methods	B12
Master most of the theoretical knowledge of course teaching	B13
Learn to analyze and solve problems independently	B14
Patiently answer students' questions	B15

**Table 2:** Comparison of the results of various indicators of different models.

Model	MAPE	MSE	SMAPE (%)	RMSE	Training time (s)
Standard-BP	0.06856	47.52	1.52	6.89	16.37
SVM	0.04725	28.37	1.15	4.59	0.326
Adaptive BP	0.04673	26.56	1.12	4.45	0.535
DDAE-SVR	0.0451	24.12	1.11	4.28	5.126

## Data Availability

The datasets used during the current study are available from the corresponding author on reasonable request.
